# Value Research of NLR, PLR, and RDW in Prognostic Assessment of Patients with Colorectal Cancer

**DOI:** 10.1155/2022/7971415

**Published:** 2022-04-16

**Authors:** Wanchen Chen, Shen Xin, Baohong Xu

**Affiliations:** Department of Gastroenterology, Beijing Luhe Hospital, Capital Medical University, Beijing 101149, China

## Abstract

**Objective:**

This study aimed to investigate the relevance of the study with the neutrophil count and lymphocyte count ratio (NLR), platelet count and lymphocyte count ratio (PLR), and red blood cell distribution width (RDW) in the prognostic evaluation of colorectal cancer patients.

**Methods:**

143 patients with colorectal cancer from January 2016 to January 2019 were selected by our hospital, and then, other 143 cases of physical examiners as normal groups were selecting to proceed colonoscopic biopsy to diagnose 106 cases of precancerous diseases related to colorectal cancer. Among them were the inflammatory bowel group (*n* = 56) and the colorectal polyp group (*n* = 50). Analysis of the survival impact factors of patients with carcinoma of the rectum, preoperative NLR, ROW, PLR, and prognostic relationship, and comparison of NLR, PLR, and RDW diagnostic rate and expression were performed.

**Results:**

Tissue type, TNM stage, lymph node metastasis, NLR, RDW, and PLR had a predictive influence on patients with colorectal cancer (*P*0.05). There was no link between gender, age, aetiology, pathological type, and prognosis in patients with colorectal cancer (*P* > 0.05). Multiple variables in patients with colorectal cancer are affected by tissue categorization (poor differentiation), TNM stages (III, IV), lymph node metastases, NLR, ROW, and PLR (*P*0.05). When compared to solo NLR, Row, and PLR diagnostics, the combination diagnosis and malignancy rates were greater, and the differences were statistically significant (*P*0.05). Diagnostic sensitivity, specificity, and accuracy were greater when compared to single NLR, ROW, and PLR. When compared to the normal control group, NLR, ROW, and PLR have greater levels, and the differences are statistically significant (*P*0.05). The patient survival declines more slowly as PLR, NLR, and the severity of the condition rises.

**Conclusion:**

NLR, ROW, and PLR combined diagnosis has high accuracy in colorectal cancer diagnosis, and the prognosis of patients with NLR, ROW, and PLR levels has a tight association; so, clinically, the above signs should be identified, and the optimal treatment time is grasped.

## 1. Introduction

The colorectal cancer is a higher incidence of malignant tumor disease. The mortality rate and incidence rate are high; therefore, the clinical exploration of effective methods diagnosis and the treatment is critical [1]. Studies have confirmed that tumor-related inflammatory cells can have a direct role in tumors and play an important role in tumor metastasis, angiogenesis, and extracellular matrix [2].

NLR and RDW can reflect the system of anti-inflammatory response, tumor presence, invasion, metastasis, and recurrence, and NLR, PLR, and clinical response to the body promoted tumor and antitumor immune response' evaluation [3]. Another scholar confirms that RDW will have significant abnormalities in malignant tumors [4]. Nevertheless, the clinical report is not much in this area; in order to investigate the prognosis of NLR, PLR, and RDW levels and the colorectal cancer patient, the study selected colorectal cancer patients, colorectal cancer-related cancer, and analyzed NLR, PLR, and RDW levels change trend, hoping to provide a theoretical foundation for disease diagnosis, and the relevant content will be reported as follows.

## 2. Data and Methods

### 2.1. General Information

From January 2016 to January 2019, 143 colorectal cancer cases in our hospital were selected and other 143 cases were selected as the normal group, and colonoscopic biopsy was selected as 106 cases of precancerous lesions are related to colorectal cancer Among them were the inflammatory bowel disease group (*n* = 56) and a colorectal polyp group (*n* = 50). 143 patients with rectal cancer, 76 males, 67 female, (53.6 ± 3.8) years old, tissue classification: 25 patients with low-differentiated patients, high, medium differential patients; onset: 45 cases of rectum, rising 39 cases of colon, 27 ethyl colon, 13 cases designed, and 19 cases. The research object agreed with the study; in the meanwhile, the research data are comparable (*P* > 0.05), and the hospital ethics committee agreed with the study. Informed consent was obtained from the patients who were participating.

### 2.2. Inclusion Criteria

1. No hypertension
2. No cellular hyperthyroidism
3. No active hemorrhage and no bleeding quality
4. Clinical data are complete and patients signed informed consent
5. No autoimmune system diseases

### 2.3. Exclusion Criteria

1. Patients with liver and kidney or cardiopulmonary function
2. Age <18-year-old patient
3. Patients with malignant tumor disease
4. Folic acid or vitamin lack patient
5. Causes straightening reactive disease

## 3. Methods

Fasting for 12 hours before detection was advised, and after extracting 3 mL of fasting venous blood, lymphocyte count, platelet count, RDW, neutrophil count, peripheral blood, and white blood cell count (Model: Beckman Cul Special LH-750) were observed. Following the completion of the detection, the PLR value is derived using the NLR and RDW detection results. Patients are followed up on for two years by WeChat, phone, and other means, and the patient's survival time is reported.

### 3.1. Observation Indicator

#### 3.1.1. Explosion Factors Affecting Rectal Cancer Patients

The explosion factors affecting renal cancer patients include gender, age, tissue classification, pathogenesis, TNM stage, pathological type, lymph node metastasis, NLR, RDW, PLR, and other factors.

#### 3.1.2. Preoperative NLR, ROW, PLR, and Prognosis

In preoperative NLR, ROW, PLR, and prognosis, add up tissue classification (low differentiation), TNM stages (III and IV), lymph node metastasis, NLR, ROW, PLR, and other factors.

#### 3.1.3. NLR, PLR, and RDW Diagnostic Rate

Calculate the calculation rate of diagnosis examples of benign and malignant patients.

#### 3.1.4. NLR, PLR, and RDW Expression

Add up 0, 20, 40, 60, and 80 months to correspond to NLR, PLR, and RDW survival rate, respectively. PLR normal range [5] is (1.5 ± 0.9), PLR >  103.7 represents the PLR abnormality; NLR normal range is (1.5 ± 0.9), NLR > 2.4 represents the NLR abnormalities; RDW normal range is (10.0 ± 2.6) FL, NLR > 12.58FL represents the RDW anomaly.

### 3.2. Statistical Method

Enter the acquired data into the Excel form, use statistics SPSS 22.0 software to perform data analysis, and conduct normal distribution inspection on the acquisition data, such as data compliance with normal distribution, count data, comparison ratio, and intergroup difference.

Using econometrics to carry out gender analysis, select card measurement. Selection card data were represented, and the differences of selection groups were analyzed. The data are represented, and the difference analysis of the group is chosen. The physical impact factor of the case group is calculated using logistic regression analysis, with a *P*value of less than 0.05 indicating that the difference is statistically significant. The image analysis software used by the Research Institute was GraphPad Prism 8.

## 4. Results

### 4.1. Prognosis Analysis of the Single Survival Factor in Patients with Colorectal Cancer

The prognosis affecting the single survival factor in patients with colorectal cancer is tissue typing, TNM stage, lymph node metastasis, NLR, RDW, PLR (*P* < 0.05), gender, age, pathogenesis, and pathological type, which has no correlation with the prognosis of patients with colorectal cancer (*P* > 0.05) (Table 1).

### 4.2. Analysis of Multifactors of Prognostic Survival in Patients with Rectal Cancer

The analysis of multifactors of prognostic survival in patients with rectal cancer is tissue classification (low differentiation), TNM stages (III and IV), lymph node metastasis, NLR, ROW, and PLR (*P* < 0.05) (Table 2).

### 4.3. Comparison of NLR, ROW, and PLR Diagnosis in Positive Rate and Malignancy

Compared with single NLR, ROW, and PLR diagnosis, combined diagnosis, positive rate and malignancy, revealed differences which have a statistical significance (*P* < 0.05) (Figure 1).

### 4.4. Comparison of NLR, Row, and PLR Diagnostic Sensitivity, Specificity, and Accuracy

Compared with single NLR, Row, and PLR diagnosis, combined diagnosis has higher sensitivity, specificity, and accuracy, and the differences have a statistical significance (*P* < 0.05) (Figure 2).

### 4.5. Comparison of NLR, ROW, and PLR Expression in Each Group

Compared to the normal control group, colorectal polyp group, and inflammatory bowel disease group, NLR, ROW, and PLR have higher levels of expression; in comparison between groups, there is a statistical significance (*P* < 0.05) (Figure 3).

### 4.6. Preoperative NLR, ROW, PLR, and Prognosis Relationship

Patient survival rates are steadily dropping as PLR and NLR levels rise in conjunction with increasingly severe conditions (Figure 4).

## 5. Discussion

The detrimental degree of colorectal cancer is severe, affecting the normal life of the patient. The current clinical research hotspot is to explore accurate diagnosis methods, improve prognosis, and reduce the degree of harm to patients [6, 7]. Several studies have proven the importance of NLR, PLR, and other markers in the prognosis of these cancers, which may be examined and monitored for systemic inflammatory response [8–10].

The study detected the value exploration of RDW, NLR, and PLR levels in colorectal carcinoma and analyzed the diagnosis, accuracy, and sensitivity. The results showed that there was a statistically significant significance for combined diagnosis and specificity and differences in combination diagnosis. The main reason is that Row is the platelet count and lymphocyte count ratio, and platelets can secrete due to secretion of P selector in adhesion, endothelial, and inflammatory cells, having promotion [11]. Platelet secretion of vascular endothelial growth factors, migration, and proliferation of endothelial cells have an induction effect, increased vascular permeability, tumor cell penetrating machine vascular metastasis, and invasive chances [12, 13]. RDW reflects the heterogeneous parameters of red blood cell size and peripheral blood [14, 15]. In addition, research shows that various factors will affect PLR and NLR individual test results and reduce sensitivity and specificity [16]. Therefore, PLR is carried out in patients with colorectal cancer, and NLR combination is very necessary. It has been shown that RDW is significantly expressed in several solid cancers, including lung cancer, breast cancer, esophageal squamous cell carcinoma, renal cell carcinoma, and other solid cancers, and that the prognosis of patients with solid tumors is closely associated with the expression of RDW [17]. Scholars pointed out that [18] tumor and PLR and NLR have a positive link with increasing NLR levels in the body, and if the number of lymphocytes is lowered, the body's immunisation balancing function will be affected, leading to tumor metastasis and proliferation. The patient's prognosis is heavily influenced by these factors. The study explores a multifactor survival in rectal cancer patients. The results showed tissue classification (low differentiation), TNM stages (III and IV), lymph node metastasis, NLR, ROW, and PLR for neutral colorectal cancer prognosis (*P* < 0.05). The main causes of RDW, NLR, and PLR affect the prognosis of colorectal cancer patients, the level of inflammatory factors increased, and the risk of colorectal cancer increased. Neutral granulocytes are N2 in the tumor state, which can pass base metal protease and vascular endothelial growth factor' effect on tumor cell apoptosis, which has promoted tumor angiogenesis, and tumor progression accelerates [19, 20]. Lymphocytes induce apoptosis of target cells, which is a tumor immune apoptotic cell, and the cytotoxic effect is obvious [21]. In addition, platelet aggregation increases the growth of tumor growth [22]. PLR and NLR are important markers for systemic inflammation and can be evaluated against inflammatory response [22]. The body's inflammatory response is raised by PLR and NLR levels, and the tissue infiltration and angiogenesis have promotion, which can cause tumor diffusion [23]. After the neutrophil is activated, the intravenous system reaches around tumor cells, the amount of active oxygen release increases, and the degree of cell DNA is damaged [24]. Therefore, it is necessary to create a microenvironment suitable for tumor cells. Tumor cell metastasis, growth, and platelet levels have significant correlation. PLR and NLR levels' increase will reduce the number of lymphocytes; the body's immunoassay is affected, and tumor cellular immunity is weakened, which is not conducive to the recovery of the condition [24]. In addition, scholars pointed out that PLR and NLR levels have correlation with patient survival. The results show that the survival time is negatively correlated with the survival rate, and the systemic inflammatory reaction equilibrium of patients with colorectal cancer is not high, which will inhibit antitumor immune response. The stage of disease and PLR and NLR have close ties with the PLR and NLR levels, which will reduce the 5-year survival rate largely. The findings revealed that single tissue type, TNM stage, lymph node metastasis, NLR, RDW, PLR (*P*0.05), sex, age, disease location, pathological type, and prognosis of colorectal cancer patients have no correlation (*P*0.05). A comprehensive analysis should influence clinical prognostic factors in patients with colorectal cancer, and targeted interventions, with individual treatment, improve patient survival. The appraised value of research was analyzed using NLR, PLR, and RDW in the prognosis of patients with colorectal cancer and higher clinical feasibility, but this study is a retrospective analysis which included a limited number of cases. The accuracy of the results will have an impact. Following that, the sample should contain more qualified individuals who do a more in-depth investigation into immune inflammation; in order to increase the accuracy of research, lengthen the lifespan of the patient and improve the patient's quality of life.

In summary, in terms of diagnosis of colorectal cancer, NLR, ROW, and PLR combined diagnosis is with high accuracy, and prognosis of patient with high NLR, ROW, and PLR levels has a close relationship; so, clinically, the above indicators should be detected and grasped for the best treatment timing.

## Figures and Tables

**Figure 1:** Comparison of NLR, ROW, and PLR diagnosis in positive rate and malignancy.

**Figure 2:** Comparison of NLR, Row, and PLR diagnostic sensitivity, specificity, and accuracy.

**Figure 3:** Comparison of NLR, ROW, and PLR expressions in each group.

**Figure 4:** Preoperative NLR, ROW, PLR, and prognosis relationship.

**Table 1:** Prognosis analysis of the single survival factor in patients with colorectal cancer.

Variables		Count	Death	Survivor	*X* ^2^/t	*P*

Gender	Male	76	37 (52.1)	39 (54.2)	0.524	>0.05
	Female	67	34 (47.9)	33 (45.8)		
Age	<65	82	34 (49.3)	48 (64.9)	0.043	>0.05
	≥65	61	35 (50.7)	26 (35.1)		
Tissue	Low differentiation	25	23 (35.9)	2 (2.5)	6.327	<0.05
	High, midphase	118	41 (64.1)	77 (97.5)		
Constraint	Rectum	45	20 (31.3)	25 (31.6)	0.728	>0.05
	Jigged	39	17 (26.6)	22 (27.9)		
	Ethyl colon	27	13 (20.3)	14 (17.7)		
	Colon	13	6 (9.4)	7 (8.9)		
	Other	19	8 (12.5)	11 (13.9)		
TNM staging	I, II	18	4 (6.3)	14 (17.7)	5.634	<0.05
	III, IV	125	60 (93.7)	65 (82.3)		
Pathological type	Aden cancer	138	61 (96.8)	77 (97.5)	1.724	>0.05
	Other (printed ring) cellular carcinoma, tubular cancer, and high-level epithelial tumor	5	2 (3.2)	2 (2.5)		
Lymph node metastasis	Yes	63	58 (92.1)	5 (6.3)	6.247	<0.05
	No	80	5 (7.9)	75 (93.7)		
NLR	—	—	5.0 ± 1.3	2.9 ± 0.6	13.854	<0.05
RDW (FL)	—	—	17.3 ± 2.2	13.9 ± 1.4	16.724	<0.05
PLR	—	—	4181.6 ± 35.8	106.3 ± 2.4	20.838	<0.05

**Table 2:** Analysis of multifactors of prognostic survival in patients with rectal cancer.

Influencing factors	B value	SE	Wald *X*^2^ value	OR value	95% CI	*P* value

Organizational profile: low differentiation	0.914	0.204	21.343	2.48	1.66–3.74	<0.001
TNM stages: III, IV	1.592	0.416	12.285	4.90	2.16–11.14	<0.001
Lymph node metastasis	0.501	0.124	19.533	1.64	1.28–2.12	<0.001
NLR	0.417	0.121	14.725	1.50	1.18–1.93	<0.001
Row (FL)	0.724	0.144	19.414	2.05	1.54–2.75	<0.001
PLR	0.711	0.313	21.545	2.02	1.09–3.78	<0.001

## Data Availability

The data used to support the findings of this study are available from the corresponding author upon request.
